The article "Extracting a Novel Emotional EEG Topographic Map Based on a Stacked Autoencoder Network" was published in 2023. Journal: J Healthc Eng.

# Extracting a Novel Emotional EEG Topographic Map Based on a Stacked Autoencoder Network

**DOI:** 10.1155/2023/9223599

**Published:** 2023-01-19

**Authors:** Elnaz Vafaei, Fereidoun Nowshiravan Rahatabad, Seyed Kamaledin Setarehdan, Parviz Azadfallah

**Affiliations:** ^1^Department of Biomedical Engineering, Science and Research Branch, Islamic Azad University, Tehran, Iran; ^2^School of Electrical and Computer Engineering, College of Engineering, University of Tehran, Tehran, Iran; ^3^Tarbiat Modares University, Tehran, Iran

## Abstract

Emotion recognition based on brain signals has increasingly become attractive to evaluate human's internal emotional states. Conventional emotion recognition studies focus on developing machine learning and classifiers. However, most of these methods do not provide information on the involvement of different areas of the brain in emotions. Brain mapping is considered as one of the most distinguishing methods of showing the involvement of different areas of the brain in performing an activity. Most mapping techniques rely on projection and visualization of only one of the electroencephalogram (EEG) subband features onto brain regions. The present study aims to develop a new EEG-based brain mapping, which combines several features to provide more complete and useful information on a single map instead of common maps. In this study, the optimal combination of EEG features for each channel was extracted using a stacked autoencoder (SAE) network and visualizing a topographic map. Based on the research hypothesis, autoencoders can extract optimal features for quantitative EEG (QEEG) brain mapping. The DEAP EEG database was employed to extract topographic maps. The accuracy of image classifiers using the convolutional neural network (CNN) was used as a criterion for evaluating the distinction of the obtained maps from a stacked autoencoder topographic map (SAETM) method for different emotions. The average classification accuracy was obtained 0.8173 and 0.8037 in the valence and arousal dimensions, respectively. The extracted maps were also ranked by a team of experts compared to common maps. The results of quantitative and qualitative evaluation showed that the obtained map by SAETM has more information than conventional maps.

## 1. Introduction

Emotion is one of the essential cognitive aspects of human beings. According to cognitive studies, evaluation of human emotion in contact with individuals and social environments plays an important role in behavior human daily life [1]. The emotion of a normal individual can be recognized by processing body reactions including facial expressions, voice, body gesture, and electrophysiological reactions. Electrophysiological signals are more preferable, especially in case of abnormal individuals, which other body reactions rarely represent internal emotional states. Therefore, the study of emotions would have a great impact on the treatment process of diseases such as depression, autism, epilepsy, and similar cases [2]. In addition, emotion recognition is an interesting topic in many research areas. The brain-computer interface (BCI) system introduces methods such as recording physiological signals from the human brain based on the central nervous system [3]. Physiological signals record the electrical activity of neurons in the brain in different parts of the cerebral cortex. Electroencephalogram (EEG), which has been used to detect brain abnormalities, is a noninvasive method for recording brain signals [4] and contains rich information about internal emotional states with the most comprehensive features. The EEG signal can be processed by the state-of-the-art marching learning methods, machine learning classifiers, and classification approach.

The article "Extracting a Novel Emotional EEG Topographic Map Based on a Stacked Autoencoder Network" was published in 2023. Journal: J Healthc Eng.

Machine learning is one of the leading methods in developing BCIs. Machine learning has many subsets such as recurrent networks, deep learning networks, and Boltzmann networks, which have their own strengths and weaknesses based on the application [1, 5, 6]. Deep learning is a specialized example of this method, which has been considered in recent decades. The development of machine learning algorithms is an interesting topic in the field of cognitive science. Deep learning networks are a trending machine learning subject capable of detecting underlying states hidden in EEG signals. Deep learning, especially in the case of large dataset such as EEG, shows acceptable and citable results in both supervised and unsupervised EEG classifications [6].

Autoencoder (AE) is a special type of artificial neural network and one of the deep learning algorithms, which automatically learn the compressed representation of raw input data [7]. Autoencoders (AEs) can extract low-level features from the input layer and high-level features in deep layers, which is well done with the structure of stacked autoencoders (SAEs) [8]. AEs extract complex nonlinear patterns from EEG data, which make the process of diagnosing and treating diseases more accurate. Zhao and He [9] developed deep learning networks to analyse early-stage Alzheimer's disease from the EEG signal and reported 92% accuracy to increase the diagnosis of this disease. Jose et al. [8] employed SAEs to study epilepsy and detected epileptic seizures by EEG signals and extracted features, such as relative energy, spectral features, and some nonlinear features from each channel. These data were imported as input to an autoencoder network, which resulted in 91.5% accuracy in the diagnosis of seizure with the concept of adaptive. Furthermore, the study of AE networks in emotion recognition from EEG data has received much attention in recent decades. Yin et al. [6] conducted studies on emotion recognition through deep networking based on a multiple-fusion-layer based ensemble classifier of stacked autoencoder (SAE). Using the AE network could increase the average classification by up to 5.26% compared to other emotion recognition networks [6]. On the other hand, the combination of neural networks is one of the most recently published for emotion classification. Liu et al. [10] combined a convolutional neural network (CNN), SAE deep neural network, and a deep neural network (DNN) to classify emotional states and reported acceptable results compared to a neural network method.

The article "Extracting a Novel Emotional EEG Topographic Map Based on a Stacked Autoencoder Network" was published in 2023. Journal: J Healthc Eng.

The EEG signal has acceptable temporal resolution and it does not provide useful information in terms of spatial resolution [11, 12]. As a result, spatial resolution of EEG contains rich information about emotional states. One of the common methods in visualizing EEG signal is quantitative EEG (QEEG) analysis, that is well known as topographic brain mapping, which provides a cost-effective and practical method for spatial evaluating of neural activities. This method represents structural and effective communication in nerve cells, nerve complexes, and brain structure [13]. Brain topography by the QEEG technique is obtained by extracting features from the EEG signal. Today, with the advancement of topographic maps, the analysis of EEG provides a comprehensive exploration of temporal and spatial characteristics simultaneously [12, 13].

In conventional “topographic brain mapping” technique, only one feature is considered to draw a map. For instance, the classical Fourier transform is calculated to quantify the power spectrum in the frequency subband of EEG signal [14], and entropy is another feature derived from EEG signal for brain mapping. Keshmiri et al. [15] examined entropy to differentiate between the brain's negative, neutral, and positive states to emotional stimuli. Moreover, power spectrum density (PSD) is another feature, which provides a separate topographic brain map [16]. As a consequence, investigating all the features underlying the EEG signal would create a larger number of topographic brain maps.

This study aimed to evaluate the hypothesis that compression of temporal, frequency, linear, and nonlinear EEG features can provide original and useful information about brain function in the form of topographic brain maps. Thus, we have presented a novel method to reduce the number of topographic brain maps to only one map by preserving spatial features and extracting the optimal combination of all features that existed in EEG signals. Therefore, the resulting topographic brain map is a specific combination of the extracted feature while preserving the spatial EEG signals features [11]. Therefore, a method is required to extract the optimal combination of EEG features. Hence, an AE-based optimal feature selection network was proposed to extract the optimal topographic brain map (stacked autoencoder topographic map-SAETM), which would provide more complete information about brain functions. In addition, evaluating one map instead of several maps speeds up the diagnostic process. To prove the study hypothesis, SAETM and conventional topographic maps were compared in a quantitative and qualitative manner. There are many common criteria for measuring the similarity of two images, including absolute error, mean square error, peak signal-to-noise ratio, histogram, similarity of Euclidean distance, or correlation coefficient to compare two independent images [17] and also using classifier methods. Accordingly, Topic and Russo [3] revealed that CNN networks have the highest performance in calculating similarity between maps of different classes. In addition, similar studies on the DEAP database by topographic brain maps with deep learning networks have enhanced the process of emotion recognition based on Capsule neural network (CapsNet) [18]. Finally, the SAETM and conventional topographic brain maps were compared by a team of specialists based on a scale questionnaire for further evaluation.

The article "Extracting a Novel Emotional EEG Topographic Map Based on a Stacked Autoencoder Network" was published in 2023. Journal: J Healthc Eng.

## 2. Materials and Methods

The study consists of four main parts, including EEG signal processing, stacked autoencoder network, emotion classification, and algorithm parameters, extracting a new topographic brain map. The first part includes EEG signal preprocessing and extraction of conventional features in emotion recognition as well. In the second part, the extracted features are abstracted by the autoencoders. The best structure of features is obtained by the emotion classifier in part three. In the last part, the ultimate features are used to draw the topographic brain map. The architecture of the SAETM is illustrated in Figure 1, including primary feature extraction (part 1), SAEs networks for abstracted feature extraction (part 2), multilayer perception (MLP) networks to extract final features based on emotion classification (part 3), and topographic brain mapping (part 4). As shown in Figure 1, the EEG signal features are extracted for each channel and fed to an SAE network. Thus, there are 32 SAE networks. At the output of each SAE, an MLP network is used to obtain a final feature; therefore, one feature is obtained for each channel. Moreover, there is an MLP classifier that is applied to the output of the previous MLPs layer. The output of this classifier is used for emotion classification, in arousal and valance dimensions, that the parameters of the SAETM algorithm will be adjusted by this classifier. A colour is assigned proportionally to each weight of the first MLPs layer to draw a topographic brain map.

The article "Extracting a Novel Emotional EEG Topographic Map Based on a Stacked Autoencoder Network" was published in 2023. Journal: J Healthc Eng.

### 2.1. Database

In this study, DEAP physiological dataset was used in emotion analysis with simultaneous recording of EEG signals and eight electrophysiological signals, including skin galvanic, respiratory rate, skin temperature, pulse rate, blood pressure, neck and smile muscle activity, and EOG signal. The EEG signal was recorded through 32 locations based on the International 10–20 system. The study was conducted on 32 healthy participants aged 19–37 (mean age 26.9), half of whom were women. This experiment was designed in a controlled environment to stimulate emotions. Forty music videos were played based on different emotional states when recording the signals. There was a 3-second interval between each music video to reset the participant's emotional states. The baseline signal was recorded for 5 seconds and after that the videos were randomly displayed to the participants. Those videos that were used as emotional stimuli were categorized with emotional labels using the self-assessment Mankins questionnaire. Then, the participant gave each video a score of one to nine after watching the full videos. Scores 1 to 3 corresponded to the negative state of the valence dimension and the inactive state in the arousal dimension, 4 to 6 were related to the neutral state of the valence dimension and the normal state in the arousal dimension, and 7 to 9 were relevant to the positive state of the valence dimension and the active state in the arousal dimension. These scores were divided into happy, pleased, relaxed, excited, neutral, calm, distressed, miserable, and depressed classes, which were related to four dimensions of emotion valence (positive/negative), arousal (passive/active), liking (like/dislike), and dominance [19].

### 2.2. Preprocessing

In the preprocessing part, unwanted noises and artifacts in the signal are removed. This study aimed to investigate electroencephalographic signals from the DEAP dataset. The 1-minute (trial) EEG signals of each video were recorded with a sampling frequency of 256 Hz and converted to a frequency of 128 Hz using the down sample method. Then, all the EEG trials were filtered to 0.05–47 Hz. Recorded EEG is affected by several noises and artefacts. The independent component analysis (ICA) algorithm extracts statistically independent components from a mixture of sources. In this study, the ICA was used to remove unwanted signals, including EMG and EOG signals. On average, 1–3 artifact-related independent components (ICs) were removed per participant.

The article "Extracting a Novel Emotional EEG Topographic Map Based on a Stacked Autoencoder Network" was published in 2023. Journal: J Healthc Eng.

### 2.3. Primary Feature Extraction

Feature selection is considered as one of the most important parts since these features can describe the signal. EEG signal features are divided into three main classes of time, frequency, and time-frequency features [11]. In this study, features, including power and statistical features as linear features and entropy, fractal dimension, and correlation dimension as nonlinear features are selected, which were considered in previous emotion recognition studies. The calculation of power is a common feature for all EEG subbands [20, 21]. Power spectrum density for five subbands, theta (4–8 Hz), low alpha (8–10 Hz), upper alpha (10–12 Hz), beta (12‒30 Hz), and gamma (30 Hz higher) is calculated by Welch's method [22]. Mean, standard deviation, and zero-crossing rate are examined as statistical features [6] and signal complexity is measured by entropy [1]. The fractal dimension is used for measuring the complexity and irregularity of the signal [23]. The correlation dimension shows the relationship between the signal and itself, which extracts repetitive and periodic patterns of the signal [24] that these features were extracted from the filtered signal. The extracted features were normalized to the baseline signal in the range of zero and one.  Table 1 lists the features extracted in this study based on previous studies [23].

All data were labelled according to the arousal-valance domain. The data labels were used for supervised training of the SAME algorithm. The trials were 1-minute intervals in which music videos with different emotional states were shown. The DEAP dataset of each trial specified a number from one to nine, which was assigned to it. This study focused on the high arousal-high valence, low arousal-high valence, high arousal-low valence, and low arousal-low valence. The reason for this choice is that the difference between the positive and negative levels of the valence scale and the high and low levels of the arousal scale are very significant. These two scales have two complementary and different aspects to examining positive and negative emotions [22]. A 2-second window with 50% overlap was used to extract the features. A total of 8 music videos were played in high arousal-high valence. 60*∗*8*∗*10 (60 windows*∗*8 music videos*∗*10 features) features were extracted from the first area. The low arousal-low valence included 12 music videos, and the extracted features were 60 windows*∗*12 music videos*∗*10 features. The two parts of low arousal-high valence and high arousal-low valence played ten music videos, 60*∗*10*∗*10 (60 windows*∗*10 music videos*∗*10 features) features were extracted for each area [19] (Figure 2).

The article "Extracting a Novel Emotional EEG Topographic Map Based on a Stacked Autoencoder Network" was published in 2023. Journal: J Healthc Eng.

## 3. Stacked Autoencoder Topographic Map (SAETM)

The autoencoder is a deep learning network to get a better description of the features [24]. Autoencoders have a symmetrical structure and the inputs and outputs are similar [7]. Each layer of autoencoders consists of three layers (input layer, one hidden layer, and one output layer). The hidden layer contains two parts, encoder and decoder. The stacked autoencoder includes several autoencoders with a SoftMax layer. The input of the first layer of the SAE network is the features extracted from the EEG signal (Table 1). These features are weights and biases calculated with the training of the first AE network. The output of the encoder at this stage is the input of the next AE network. This process continues to obtain the final abstracted features, and finally, the output of the last AE network encoder is used to classify emotions [25].

In the first step of the SAEs training, the network uses unlabelled data to extract EEG abstracted features in an unsupervised procedure. Then, the encoder part is completed with a classifier and it trained with supervised procedure to finetuning the SAE parameters. It can help to initialize the weights one layer at a time by minimizing the reconstruction loss.

Assuming that the vector of the extracted features from input and the vector of the hidden layer are *x* ∈ R^*n*^ and *h* ∈ *R*^*m*^, respectively, *n* is the dimension of the extracted features in input and *m* is the dimension of abstracted features (Equation (1)) (*R* is real number).

(1) $$\begin{array}{c} h=\sigma \left(x.W+b\right), \end{array}$$

where *W* ∈ *R*^*m*×*n*^ is a weight matrix, *b* ∈ *R*^*m*^ is a bias vector, and *σ* is an activation function (sigmoid function) (Equation (2)) that is located in the output layer.

(2) $$\begin{array}{c} \sigma \left(z\right)=\frac{1}{\left(1+e^{-z}\right)}\text{.} \end{array}$$

x′ ∈ *R*^*n*^ is the next layer that has the same dimension as the input vector. The output reconstructs the input vector by updating the hidden layer weights.

(3) $$\begin{array}{c} x\prime =\sigma \left(h.W^{T}+c\right)\\ =\sigma \left[\sigma \left(x.W+b\right).W^{T}+c\right]\text{.} \end{array}$$

The autoencoder parameters, *W*, W^*T*^, *b*, and *c* are obtained by the backpropagation algorithm by the square error cost function according to equation (4) that *l* is considered the number of the training samples.

(4) $$\begin{array}{c} E=\overset{l}{\underset{k=0}{\sum }}{\left(x-x\prime \right)}^{2}\text{.} \end{array}$$

The next autoencoder layer is used by *h* and this operation is repeated *l* times to produce a stacked autoencoder. The best abstracted features are produced in the hidden layer of each autoencoder and *h*^(*l*)^ is the best representation of abstracted features (Equation (5)).

(5) $$\begin{array}{c} h^{\left(l\right)}=\sigma \left(W^{\left(l\right)}\cdots \sigma \left(W^{\left(2\right)}\sigma \left(W^{\left(1\right)}x+c^{\left(1\right)}\right)+c^{\left(2\right)}\right).+c^{\left(l\right)}\right)\text{.} \end{array}$$

This stage is called pretraining to set SAE parameters. An MLP network with one output neuron is added to the encoder side of each SAE to extract the one abstracted feature in order to plot brain map in topographic map stage. *U*^*i*^ is the output function in which µ is the matrix of weights and *∂* is the bias vector in the MLP layer, and *i* is the number of SAEs.

(6) $$\begin{array}{c} U^{i}=\sigma \left(µh^{\left(l\right)}+\partial \right)i\in \left\{1,2,\text{..}32\right\}\text{.} \end{array}$$

The feature sets are defined as *F*^(*n*)^. It means that the features of each channel are grouped into ten parts, the power is *F*_1_, *F*_2_, *F*_3_, *F*_4_ (four subbands are selected). The linear EEG features including means, standard deviation, and zero-crossing rate are *F*_5_, *F*_6_, and *F*_7_, respectively. In the end, *F*_8_, *F*_9_, and *F*_10_ are built based on nonlinear features, fractal dimension, approximate entropy, and correlation dimensions. Therefore, feature vectors are defined, x(*F*_*j*_) ∈ *F*_*j*_ , *j* ∈ {1,2, .10}. We construct *i* SAE for describing the hidden feature abstractions of each channel based on equation (7), where *S*_sae_^1^(x),… *S*_sae_^32^(x) denote the higher feature abstractions of each channel features.

(7) $$\begin{array}{c} \left\{\begin{array}{l} U^{1}=\sigma \left(µh^{\left(l\right)}+\partial \right)=S_{sae}^{1}\left(x\right)\text{,}\\ U^{2}=\sigma \left(µh^{\left(l\right)}+\partial \right)=S_{sae}^{2}\left(x\right)\text{,}\\ \ldots \\ U^{32}=\sigma \left(µh^{\left(l\right)}+\partial \right)=S_{sae}^{32}\left(x\right)\text{.} \end{array}\right. \end{array}$$

The structure of the SAETM is completed by placing two neurons in the last layer (Equation (8)), where $y=\left(\begin{array}{c} 1\\ 0 \end{array}\right)$ or $y=\left(\begin{array}{c} 0\\ 1 \end{array}\right)$ shows the low and high levels of emotion dimensions.

(8) $$\begin{array}{c} y=\sigma \left(\beta U^{i}+\alpha \right)\text{.} \end{array}$$

where *y* is the output function in which *β* is the matrix of weights and *α* is the bias vector in the last layer. The finetuning stage is an important stage of SAE networks. The finetuning method is used to train large labelled data and can improve classifier performance [6, 25]. This stage finetunes the parameters of the last layer of SAE by backpropagation algorithm in the form of training with the supervisor. The parameters obtained in part 4 are used for the topographic brain map.

The article "Extracting a Novel Emotional EEG Topographic Map Based on a Stacked Autoencoder Network" was published in 2023. Journal: J Healthc Eng.

The number of layers and the number of neurons in each SAE layer are important in SAETM training. Therefore, the minimum hidden layer and minimum number of neurons in each layer are essential for having an optimal classification. In this study, Pearson or Spearman correlation coefficients were used to find the most optimal structure [6, 10]. These two coefficients calculate the best similarity between input and output data. These two parameters calculate the best similarity between input and output data. Therefore, the structural loss function (SLF) is defined based on equation (9).

(9) $$\begin{array}{c} SLF=\omega_{1}\left(1-\rho_{1D_{x}D_{z}}^{2}\right)+\left(1-\omega_{1}\right)\left(1-\rho_{2D_{x}D_{z}}^{2}\right)\text{,} \end{array}$$

where *ω*_1_=0.5, *ρ*_1*D*_*x*_*D*_*z*__, and *ρ*_2*D*_*x*_*D*_*z*__ are the Pearson correlation coefficient and Spearman rank correlation coefficient, respectively [6], where *D*_*x*_ is the input matrix and *D*_*z*_ indicates the output matrix.

### 3.1. Classifier Evaluation

Depending on literature [26], choosing the type of classifier can affect the results. For this purpose, referenced classifiers will be used in this study and the desired classifier will be selected based on the results. To check the accuracy of the network, we consider a criterion as described below. The following equations are used to evaluate the precision of classifier of emotion classes in equation (10), in which TP is true positive and FP is false positive [27].

(10) $$\begin{array}{c} Precision=\frac{TP}{TP+FP}\text{.} \end{array}$$

The network accuracy is calculated by equation (11), where FN is a false negative.

(11) $$\begin{array}{c} Recall=\frac{TP}{TP+FN}\text{.} \end{array}$$

The classifier accuracy is generally obtained from equation (12) in which TN is true negative.

(12) $$\begin{array}{c} overall\;classification\;accuracy=\frac{\left(TN+TP\right)}{\left(TN+FN+TP+FP\right)}\text{.} \end{array}$$

The *F*1 is a combination of the accuracy and recall criteria, which is obtained according to equation (13).

(13) $$\begin{array}{c} F1\;score=\frac{2\times \left(Precision\times Recall\right)}{Precision+Recall}\text{.} \end{array}$$

The article "Extracting a Novel Emotional EEG Topographic Map Based on a Stacked Autoencoder Network" was published in 2023. Journal: J Healthc Eng.

### 3.2. Evaluating the Topographic Brain Maps

Extracting topography or brain map is one of the practical methods of QEEG. Parameters of making the brain topography are calculated for different subbands of EEG signal for each number of electrodes according to the standard of the 10–20 international system. The extracted features in the previous section are considered as colour mapping parameters. The bilinear interpolation method is used for navigating the values between the electrodes [13, 27]. In this study, the brain topographic map was extracted by the MNE library in Python software.

### 3.3. The CNN Used in Image Classification

The convolutional neural network (CNN) is a feed-forward neural network, in which the input of this network is image-like. CNNs are originally designed for evaluating images [3]. In this study, we use CNN accuracy as criteria to measure similarity between two groups of topographic maps. The building blocks in CNN architecture include convolution layer, pooling layer, and fully connected layers. The convolutional layer is the central part of a CNN. In this layer, there are multiple filter slides (or Kernel) that convolves across the input with the convolution operation. This operation has the ability to extract features with preserving spatial information from the database and the pooling layer can decrease the spatial dimension of features. In addition, the pooling layer also filters out noise from the image. An image is convolved with a filter to learn one feature from the whole image. The fully connected layers connect inputs in the previous layer, pooling layer, to the output neurons [3, 28]. Suppose a *M* × *M* image convolves with a *k* × *k* kernel. Equation (14) shows the size of the output image without padding and equation (15) is the convolution operation. Padding is used in order to preserve the size of input image. The size of the output image with padding is shown in equation (16).

(14) $$\begin{array}{c} M\times M*k\times k=M-K+1\text{,} \end{array}$$

(15) $$\begin{array}{c} O=\delta \left(B+\overset{2}{\underset{i=0}{\sum }}\overset{2}{\underset{j=0}{\sum }}w_{i,j}h_{a+i,b+j}\right)\text{,} \end{array}$$

(16) $$\begin{array}{c} M\times M*k*k=\frac{\left(M+2P-F\right)}{\left(s+1\right)}\text{,} \end{array}$$

where *O* is the output, *P* is the padding, *s* is the stride, *b* is the bias, *δ* is the sigmoidal activation function, *δ* is a 3 × 3 weight matrix of shared weights, and *h*_*x*,*y*_ is the input activation at position *x*, *y* [29].

CNN model, which is used in this study, is presented in Figure 3. Max pooling were applied as pooling method. In max pooling, the maximum activation output is pooled into a 2 × 2 input region and the parameters of the model were set as follows: Number of epochs: 10, optimizer: RMS prop, learning rate = 0.001, the parameter *β*: 0.9, activation: sigmoid, stride: 1 for convolution layer, stride: 2 for pooling layer.

The article "Extracting a Novel Emotional EEG Topographic Map Based on a Stacked Autoencoder Network" was published in 2023. Journal: J Healthc Eng.

## 4. Results and Discussion

### 4.1. Results

In this section, the results obtained from the SAETM were presented to extract topographic brain maps. The data were divided into train and test groups to evaluate this algorithm. All data were normalized for each participant with a mean of zero and a standard deviation of one to eliminate the difference in the scale of features. K-fold cross-validation method was used to evaluate the studied samples better. *k* = 10 was considered so that each time 0.1 of the data is selected for testing and trained with 0.9 of the data. This operation is repeated ten times to observe all the data by the network.

### 4.2. Architecture of the SAETM

The appropriate selection of SAETM parameters, that is, the number of hidden layers and the number of neurons in each layer, improves network performance.  Figure 4 illustrates the SLF based on (7) for the ten features selected in Table 1. The SLF was used to optimize the number of neurons in each layer that was calculated by adding the number of neurons in each layer.  Figure 4(a) represents the trend of feature abstraction in the F3 channel as an example of channels in the left hemisphere. As shown, the input of the first hidden layer is ten features extracted from the EEG signal. The SLF value has its lowest value in the first layer with seven neurons. Therefore, seven abstracted features were obtained in the first layer. Adding another neuron to this layer increases the amount of SLF. Therefore, the minimum amount of SLF, which is seven neurons in the first hidden layer, is important. The seven features extracted from the first hidden layer are the inputs of the second hidden layer. The minimum amount of SLF is observed in the second hidden layer with four neurons. Thus, ten neurons are reduced to seven neurons and finally to four neurons.  Figure 4(b) presents these calculations in the right hemisphere for the F4 channel. In this channel, ten features were reduced to six in the first hidden layer, three features in the second layer, and finally to one feature.  Figure 4(c) is similarly calculated for the Cz channel. As shown, ten features were decreased to seven features in the first layer and three in the second layer.  Table 2 shows the number of neurons in each hidden layer in each of the 32 channels. The maximum and minimum neurons in the last layer are four and one, respectively.

The article "Extracting a Novel Emotional EEG Topographic Map Based on a Stacked Autoencoder Network" was published in 2023. Journal: J Healthc Eng.

### 4.3. Accuracy Measures for the Comparison of Classifiers

The abstracted features are obtained in the last layer after finetuning the SAE parameters. According to the hypothesis of this study, the output of each SAE is used as an optimal feature to extract the brain topographic map. The performance of the SAETM algorithm was compared with several emotion classifiers.  Figure 5 demonstrates the comparison of the accuracy of emotion classifiers with the accuracy of the SAETM. KNN (K-nearest neighbour classifier), BN (naive Bayesian classifier), and SVM (support vector machines) are selected for the reason that these classifiers are known as widely used classifiers in emotion recognition field using EEG information [23].

In Figure 5, the SAETM is made up of the MLP network (multilayer perceptron) [26]. Figures 5(a) and 5(b) show the accuracy of the classifiers in the valence and arousal dimensions, respectively. The accuracy of the SAETM and SVM networks are close to each other and average accuracy of SAETM and SVM networks are as much as in the valence dimension 83.3% and 82.7% and in the arousal dimension 82.8% and 74.8%, respectively. KNN and BN networks show the average accuracy equal to in the valence dimension 74.3% and 79.2% and in the arousal dimension 73.4% and 77.2%, respectively. The SAETM method had the highest and the KNN network had the lowest accuracy. There is a significant difference between these two classifiers SAETM and SVM (*p* >  0.01) and other classifiers. The loss of the proposed SAETM structure with respect to check the generalization of this network is presented in Figure 6. As shown, the SAETM has appropriate generalization on validation data and the maximum epoch is considered 200.

Figure 7 shows a comparison of network performance with the Box–Whisker display in two dimensions, arousal (b) and valance (a). Each column corresponds to a classifier. The highest accuracy is related to SVM and MLP classifiers. The MLP network was used for simplifying the structure of the SAETM. The classification accuracy and the needed computational time for training an emotion recognition network are significant factors for building a new network structure. The computational time taken by the SAETM, SVM, KNN, and BN networks for training are illustrated in Figure 8. The BN has the highest computational time, while the KNN has the lowest value. The SAETM reports less computing time than the BN and it is near to SVM.

### 4.4. Comparison of Different Feature Extraction Methods

In this study, the SAE network was selected as the feature extraction method. The SAE network was compared with PCA feature extraction method, nonlinear PCA method, and KLDA method to evaluate the selected feature extraction method.  Figure 9 indicates the comparison of the classifier results for the 32 participants based on these three methods in the valence and arousal dimensions.  Figure 9(a) demonstrates the Box–Whisker diagram of the results of comparing SAE networks in the valence dimension, and Figure 9(b) presents its arousal dimension with PCA, nonlinear PCA, and KLDA. Linear PCA method with an average accuracy of 75.3% in the valence and KLDA method with 73.2% in the arousal dimensions reported the least accuracy, and the SAETM reported 83.3% and 82.8% accuracy in both valence and arousal dimensions, respectively. Based on the results, SAE network has better performance compared to other networks (*p* < 0.01). Computational time for training the network with different feature extraction method is shown in Figure 10. The highest value is related to KLDA method and the SAETM had the lowest computational time.

The article "Extracting a Novel Emotional EEG Topographic Map Based on a Stacked Autoencoder Network" was published in 2023. Journal: J Healthc Eng.

Some linear and nonlinear features of the EEG signal were used based on Table 1 in the designed SAETM algorithm. The three modes were examined to evaluate the selected features. In the first state, the network only trains with linear features. The second state is the desired nonlinear features, and in the third state, the combination of linear and nonlinear features was evaluated. If the input of SAE networks was linear features, the accuracy of the network in the valence and arousal dimensions is 65.7% and 64.2%, respectively. The network accuracy is 53.6% and 54.9%, respectively, by applying nonlinear features. The accuracy of the network according to Figure 5 in the valence and arousal dimensions is 83.3% and 82.8%, respectively, if linear and nonlinear features are applied as inputs to SAE networks (SAETM). In addition, the *F*1 score for the SAETM in the valence and arousal dimensions, which is obtained from equations (11) and (12) (Precision and Recall concepts) is 81.8% and 80.3%, respectively, and the SVM network is 78.4% in the valence dimension and 72.7% in the arousal dimension. Therefore, using linear and nonlinear features together gives better results than the other two modes.

### 4.5. Comparisons for Combination of Classifiers and Feature Extraction Methods

The result of accuracy comparison and computational time to combine common classifiers and feature extraction methods is shown in Tables 3 and 4 respectively, and it is visible that the accuracy of combination of SVM classifier and NPCA feature extraction method in valance (78.04), and SVM classifier and KLD method in arousal (78.23) perform better than comparable methods reported (Table 3). On the other hand, computational time to train in valence and arousal space show that the combination of the KNN classifier and PCA feature extraction method, in the valence (452 seconds) and in the arousal (470 seconds), provides less computational time in comparison with others (Table 4).

The article "Extracting a Novel Emotional EEG Topographic Map Based on a Stacked Autoencoder Network" was published in 2023. Journal: J Healthc Eng.

### 4.6. Emotional Topographic Brain Mapping

In this study, a brain topographic map is extracted by selecting the MLP network and assigning a colour appropriate to the weight of each node in this network (Figure 1). Figures 11(a) and 11(b) show the map use of the SAETM method and the common method for ten features of Table 1 while watching emotional video clips. Images obtained from sub-band power, mean, standard deviation, zero-crossing rate, fractal dimension, entropy, and correlation dimension features are observed separately in four emotion classes. The right column in Figures 11(a) and 11(b) is the images from the SAETM algorithm. The SAETM in four scales of high arousal-high valence, low arousal-high valence, high arousal-low valence, and low arousal-low valence, could create more separation for the border of active areas in the brain compared to common methods. Dark red shows the most brain activity and dark blue the least brain activity (Figure 11). In high arousal-high valence (1) in both Figures 11(a) and 11(b), the active regions in the frontal section are only in theta power and standard deviation and the images related to the two features of mean and zero-crossing rate are observed in the occipital region. Brain activity was high at relative entropy in the center of the head toward the frontal lobe. Brain activity in the three images was related to features such as theta power, relative entropy, and fractal dimension in the lower right hemisphere. Moreover, the images of relative entropy and correlation dimension in the left hemisphere indicate the lowest values of low brain activity. In the SAETM, the brain's activity in the frontal areas in the left hemisphere can be observed, along with its inactivity in the right hemisphere. The active and inactive parts are separated from the center of the head and divided into right and left hemispheres. Most of the brain activity is in the left hemisphere towards the frontal. In low arousal-high valence (2), the active part of the brain is observed in the center of the head toward the left hemisphere in images of theta, alpha, gamma, and standard deviation. The active part of the image has the maximum value of the beta power in the center of the head towards the frontal. The occipital section is neutral or inactive in all images (2) except the correlation dimension image. In the next image, the correlation of the left hemisphere shows the highest brain activity at this scale. In the SAETM image, the frontal area shows the inactive areas of the brain at this scale and the head-to-back center bar shows the active area of the brain. In this network, the image is divided into two inactive and active parts from the middle of the head into two parts, including the front and the central bar of the head, respectively. In high arousal-low valence (3), the active parts in the images are theta, alpha, beta power, and mean in the frontal region to the right hemisphere. Images of zero-crossing rate and to some extent, the fractal dimension features show the highest brain activity in the right hemisphere. The central area to the back of the head shows the activity of the brain at its lowest state in all images except the entropy feature. In the SAETM algorithm, the active and inactive parts of the brain are divided from the center of the head into right and left hemispheres. In this image, the frontal region is obtained in two fully active hemispheres. Finally, in low arousal-low valence (4), the frontal to central part of the head showed low brain activity in all images except alpha power and fractal dimension. Three images of beta power, mean, and fractal dimension in the occipital region show brain activity. In the image of the SAETM, two active and inactive parts are divided from the center of the head to the front and back of the head, which shows the brain's activity in the occipital.

The article "Extracting a Novel Emotional EEG Topographic Map Based on a Stacked Autoencoder Network" was published in 2023. Journal: J Healthc Eng.

### 4.7. Comparison of the Resulting Topographic Maps

There are several methods as numerical criteria rubric to compare the resulting topographic maps including the use of classifier networks and comparing network accuracy as a criterion for distinguishing network inputs (input images).  Table 5 shows the results of using successful networks in image classification. As shown, the map classification results of the SAETM algorithm have the highest accuracy (0.8305 ± 0.02). In addition, the average accuracy of different classifications on the images obtained from this network has the highest value (0.7613 ± 0.04). In the SAETM, the BN classifier has the lowest accuracy, which is equal to 0.6906 ± 0.12. This value is still higher than the average accuracy of the various classifiers and the average accuracy for the alpha power is 0.5863, which is the highest accuracy after the SAETM. Therefore, the images obtained by the SAETM have more distinction than any of the common images. The results obtained by Chao et al. [18] reported accuracy results as much as 0.6673 in the valence dimension and 0.6828 in the arousal dimension by creating an image by mapping the electrodes on a two-dimensional matrix. Topic and Russo [3] evaluated the images obtained from CNN network on DEAP data and extracted features from the resulting images with an accuracy of 0.7630 in the valence dimension and 0.7654 in the arousal dimension. The SAETM achieved accuracy of 0.8173 in the valence dimension and 0.8037 in the arousal dimension by CNN classification. In addition, the F1 score criterion for the SAETM in two dimensions of valence and arousal was 0.8031 and 0.7984, respectively.

The article "Extracting a Novel Emotional EEG Topographic Map Based on a Stacked Autoencoder Network" was published in 2023. Journal: J Healthc Eng.

Table 6 demonstrates the accuracy of the CNN classification after watching ten music videos. The accuracy of the CNN classification was 0.4874 after watching the first video for SAETM. The resulting image reported accuracy of 0.7923 after five minutes and 0.8305 after ten minutes. According to Table 6, CNN network classified the image from the SAETM after watching the fifth music video with the accuracy close to watching the tenth music video. Therefore, the SAETM produced a brain topographic map in a shorter time. The best accuracy was obtained in the ninth or tenth minute in CNN network accuracy for ten other features during this time.

### 4.8. Quality Evaluation of the Resulting Maps

To evaluate the quality of the resulting maps, 20 experts in the field of topographic brain maps were asked to give a score of zero to ten via scale questionnaire to EEG maps extracted from the SAETM and maps obtained from the common methods. The scale questionnaire is designed based on the rate of differentiation and meaningfulness of the photos. The results of ANOVA test show that topographic maps obtained from SAETM are preferable to common methods (*P*  < 0.001) (Figure 12). The resulting maps well differentiate the active areas in different parts of the brain while watching music videos from the rest time. Moreover, these maps show that the extracted topographic maps have spatial, temporal, and frequency information that would lead to more understanding of anatomical brain function. Therefore, topographic images, which contain rich spatial and functional information about the brain, will lead discover more implications about humans.

All software implementations were run on a Windows 10 64-bit workstation with an Intel Celeron 2.4 GHz and 4 GB of RAM.

## 5. Discussion

Electroencephalographic methodological issues have a high temporal resolution but low spatial resolution for locating the source. The sensitivity of spatial resolution decreases as a function of the depth of neural sources. Therefore, the ability to detect deep brain generators that are vital to the production of emotions is still a matter of debate. Numerous EEG studies on emotion support the idea that the impact of deep sources such as the hippocampus, the amygdala, or basal ganglia can be reasonably determined despite relatively low signal strength using a variety of source analysis methods [30].

The article "Extracting a Novel Emotional EEG Topographic Map Based on a Stacked Autoencoder Network" was published in 2023. Journal: J Healthc Eng.

Due to the fact that in the generate of emotions, the EEG signal indicates the trigger of the deeper sources of the brain, topographic brain mapping as a feasible method allows us to study emotion with more details about the activity of brain areas. In our study, the features obtained for topographic mapping are a nonlinear combination of features used in conventional brain mapping. Therefore, the only common feature of the obtained map and common maps is the degree of participation of each area of the brain in emotional activity. To compare the obtained map with common maps, we investigate the degree of participation of brain areas in different emotions. There are several studies that show stimuli with relative valence affect the interhemispheric asymmetry within the prefrontal cortex [31], which results the development of the “hemispheric valence hypothesis” [32] and it states that high valence emotions are largely processed in the left frontal cortex and low valence emotions are largely processed within the right prefrontal cortex [33].

As it can be seen in Figures 11(a) and 11(b), SAETM map is clearly interhemispheric asymmetric and shows that arousal is associated with brain activity in the right posterior cortex and valence is associated with brain activity in the left frontal lobe, which is supported by Rogenmoser et al. [34]. The relative differences in interhemisphere asymmetry between high and low valence conditions, were investigated and the results of Kolmogorov–Smirnov (ks) tests show significant differences (*p* < 0.01). We also investigate the dynamics of interhemisphere asymmetry by applying the Shannon entropy of the extracted maps (10 minute) for different valence in trials. A significant difference was found (*p* < 0.01). The results show interhemisphere asymmetry reflects activity in subcortical brain regions. Specifically changes in prefrontal asymmetry are known to be related with amygdala and cerebellum. As the SATEM map shows frontal asymmetry is well reflected in high valence-high arousal condition as well as supported by Hamann [30]. As depicted in last row of Figure 11, in low arousal-low valence condition, asymmetry relates to frontal-occipital and it can be most likely related to visual processing activity rather than emotional activity. Furthermore, this can be observed in high valence-low arousal, however, frontal asymmetry is also observed to some extent. Therefore, we can conclude that low arousal stimuli do not cause great deal of frontal asymmetry. In addition, as can be seen in high-arousal stimuli, SAETM map is asymmetric in left and right hemispheres.

The article "Extracting a Novel Emotional EEG Topographic Map Based on a Stacked Autoencoder Network" was published in 2023. Journal: J Healthc Eng.

According to the results, the following items were evaluated to test the hypotheses of this study.

- SAE networks can extract deep features in the EEG signal due to their deep structure. Feature extraction by SAE networks was compared with PCA, nonlinear PCA, and KLDA feature extraction methods. The results showed that SAE networks can extract features with the accuracy of 83.3% and 82.8% in the valence and arousal dimensions, respectively.
- The use of linear and nonlinear features was expected to provide better representations of the signal to the classifier due to the nonlinear nature of the EEG signal. The accuracy of the network was evaluated in three modes of using only linear features, nonlinear features, and finally the use of linear and nonlinear features, according to which the choice of linear and nonlinear features increased the accuracy of the network.
- The optimal number of neurons in each hidden layer for each SAE network was calculated based on the SLF. For example, ten extracted features are compressed into seven and finally into four features in the F3 channel.
- The accuracy of the SAETM for classifying the four classes of emotions is a parameter for evaluating the choice of feature extraction method. SAE networks can correctly select features due to their deep structure and the accuracy calculated in the valence dimension (83.3%) and in the arousal dimension (82.8%).
- Extracting the topographic maps of the SAETM was used in this study and the results were compared quantitatively and qualitatively with common maps. The accuracy of maps classifiers as a criterion for quantifying image differentiation indicated that CNN has the highest accuracy on maps from the SAETM (0.8305 ± 0.02). Qualitative evaluation of maps by the experts showed that maps obtained from the SAETM are significantly different from common maps.
- Features extracted from the SAETM produced maps in less time than a single feature. CNN classified maps with more than 79% accuracy five minutes after the signal. This result showed that the speed of user recognition increases by enhancing speed of image production.

Finally, the limitations in current work and further work may include the following:

- The SATEM emotion classifier presents in this study is designed by the classifier paradigm. In future studies, we propose that the network structure of the SAE be formed in an automatic manner, as well as the network structure based on the criteria and quantitative methods for generating topographic maps with the highest distinction.
- The performance of the SATEM has been undermined when data are limited. The potential reason is that the deep models require large size of data samples. On the other hand, considering that stacked autoencoders have the ability to extract deep features in the data, it is suggested to use raw EEG signal instead of the features that used in this study for SAE input to retain the spatial characteristics of EEG signals as much as possible.
- Since topographic maps provide rich information in the diagnosis of mental disorders, other directions deserving of exploration in future works include implemented on more datasets especially for mental disorders and functional network analysis based on the decoded hidden features. Moreover, the authors suggest the simultaneous fMRI and EEG to investigate the relationship between the obtained maps and the deeper sources of the brain.

The article "Extracting a Novel Emotional EEG Topographic Map Based on a Stacked Autoencoder Network" was published in 2023. Journal: J Healthc Eng.

## 6. Conclusions

In this study, we proposed and implemented a stacked autoencoder network, which creates novel emotional topographic EEG brain maps. This deep learning approach aimed to extract EEG maps with higher differentiation than common maps. This method combines EEG features commonly used in emotion studies to extract richer features in a supervised emotion classification framework. In addition, the accuracy of the classifier was considered as a criterion for optimal feature combination. Therefore, the obtained map is considered as the optimal map in terms of differentiating between different emotional states. Performance of the algorithm was approved by the quantitative and qualitative evaluation of classifier accuracy and emotional EEG maps extracted from DEAP database. The results obtained in this study show that the proposed method has an acceptable ability to create topographic brain maps with more differentiation than conventional EEG maps. It also allows us to better understand the involvement of different areas of the brain in emotional activities with the state-of-the-art deep learning models.

## Figures and Tables

**Figure 1:** Architecture of the stacked autoencoder topographic map (SAETM) algorithm.

**Figure 2:** Arousal- and valence-based emotion model. Four areas of the model are presented by the extracted features.

**Figure 3:** CNN model to classify the topographic maps.

**Figure 4:** SLF changes for the number of neurons in each layer: (a) the number of neurons in each hidden layer in the F3 channel in the left hemisphere, (b) the number of neurons in each hidden layer in the F4 channel in the right hemisphere, and (c) the number of neurons in each hidden layer in the Cz channel in centre of the head.

**Figure 5:** Comparison of emotion classifiers with SAETM for two dimensions of valence (a) and arousal (b).

The article "Extracting a Novel Emotional EEG Topographic Map Based on a Stacked Autoencoder Network" was published in 2023. Journal: J Healthc Eng.

**Figure 6:** The loss of the SAETM structure with the increase in the number of training epochs.

**Figure 7:** Box–Whisker diagram to compare SAETM classifier with SVM, KNN, and BN networks for two dimensions of valence (a) and arousal (b).

**Figure 8:** Computational time (s) to train networks.

**Figure 9:** Box–Whisker diagram to compare SAE method for feature extraction with NPCA, KLDA, and PCA methods in two dimensions of valence (a) and arousal (b).

**Figure 10:** Computational time (s) to train for different feature extraction method.

**Figure 11:** (a) Images obtained from ten features extracted from EEG signal (power for four sub-bands and mean) and images obtained from SAETM during viewing ten music videos. (b) Images obtained from ten features extracted from EEG signal (standard deviation, zero-crossing rate, fractal dimension, entropy, and correlation dimension) and images obtained from SAETM during the viewing period of ten music videos.

**Figure 12:** Statistical comparison of scores obtained from scale questionnaire for maps extracted from SAETM, EEG power sub-bands (theta, alpha, beta, gamma), mean, standard deviation (Std), zero-crossing rate (ZCR), fractal dimension (FD), approximate entropy (ApEn), and correlation dimension (CD) by ANOVA test.

**Table 1:** Features extracted in the SAETM algorithm.

Channels	Features	Formula	Feature index
Fp1, AF3, F3, F7, FC5, FC1, C3, T7, CP5, CP1, P3, P7, PO3, O1, Oz, Pz, Fp2, AF4, Fz, F4, F8, FC6, FC2, Cz, C4, T8, CP6, CP2, P4, P8, PO4, and O2	EEG power of sub-bands: Theta (4–8 Hz), alpha (8–12 Hz), beta (12–30 Hz), gamma (30–45 Hz)-average PSD	*P*=1/*N*∑_*i*=1_^*N*^|*x*_*i*_^2^|	No. 1–128 (4 features *∗* 32 channels)
		Form a time series of data *x*_*i*_=[*x*_1_, *x*_2_, ⋯, *x*_*N*_]	
	Mean	*μ*=1/*N*∑_*i*=1_^*N*^*x*_*i*_	No. 129–321 (6 features *∗* 32 channels)
		Form a time series of data *x*_*i*_=[*x*_1_, *x*_2_, ⋯, *x*_*N*_]	
	Standard deviation	*σ* ^2^=1/*N* − 1∑_*i*=1_^*N*^(*x*_*i*_ − *μ*)^2^	
		Form a time series of data *x*_*i*_=[*x*_1_, *x*_2_, ⋯, *x*_*N*_]	
	Zero-crossing rate	ZCR=1/2*N*|sgn[*x*(*n*)] − sgn[*x*(*n* − 1)]|	
		Form a time series of data *x*_*i*_=[*x*_1_, *x*_2_, ⋯, *x*_*N*_]	
	Fractal dimension	*N*=*ε*^−*D*^ where the variable *N* stands for the number of measurement units, *ε* for the scaling factor, and *D* for the fractal dimension	
	Approximate entropy	1: Form a time series of data *x*_*i*_=[*x*_1_, *x*_2_, ⋯, *x*_*N*_]	
		2: Form a sequence of vectors *U*_*j*_=[*x*_*i*_, *x*_*i*+1_, ⋯, *x*_*i*+*m*−1_] for fix *m* and real number *r*	
		3: Use the sequence *x*_*i*_=[*x*_1_, *x*_2_, ⋯, *x*_*N*−*M*+1_] to construct, for each *i*, 1 ≤ *i* ≤ *N* − *m*+1	
		*C*_*i*_^*m*^(*r*)=(number of(*x*_*j*_)such that*d*|*x*_*i*_ − *x*_*j*_| ≤ *r*)/(*N* − *m*+1)	
		4: $\varphi^{m}\left(r\right)={\left(N-m+1\right)}^{-1}\overset{=\left(N-m+1\right)}{\underset{i=1}{\sum }}\log\;\left(C_{i}^{m}\left(r\right)\right)$	
		5: ApEn = *φ*^*m*^(*r*) − *φ*^*m*+1^(*r*)	
	Correlation dimension	For any set of *N* points in an *m*-dimensional space	
		1 : *x*_*i*_^→^=[*x*_1_(*i*), *x*_2_(*i*), ⋯, *x*_*N*_(*i*)]	
		$2:C\left(\epsilon \right)=\lim_{n⟶\infty }{\left(g/N^{2}\right)}^{n}$ where *g* is the total number of pairs of points, which have a distance between them that is less than distance *ϵ*	
		3 : *C*(*ϵ*) ~ *ϵ*^*CD*^	

The article "Extracting a Novel Emotional EEG Topographic Map Based on a Stacked Autoencoder Network" was published in 2023. Journal: J Healthc Eng.

**Table 2:** Number of neurons in each hidden layer for 32 SAEs equivalent to 32 channels.

SAEs	*Hidden layer*			SAEs	*Hidden layer*		
	Hidden layer 1	Hidden layer 2	Hidden layer 3		Hidden layer 1	Hidden layer 2	Hidden layer 3
SAE (Fp1)	8	5	3	SAE (Fp2)	6	4	1
SAE (AF3)	8	4	2	SAE (AF4)	6	4	4
SAE (F3)	7	4	4	SAE (Fz)	7	5	4
SAE (F7)	6	5	2	SAE (F4)	6	3	1
SAE (FC5)	8	6	3	SAE (F8)	7	5	3
SAE (FC1)	5	4	1	SAE (FC6)	7	4	3
SAE (C3)	7	4	3	SAE (FC2)	5	3	1
SAE (T7)	5	3	3	SAE (Cz)	7	3	3
SAE (CP5)	6	4	1	SAE (C4)	6	4	2
SAE (CP1)	8	5	4	SAE (T8)	6	4	4
SAE (P3)	7	3	3	SAE (CP6)	8	4	3
SAE (P7)	7	4	2	SAE (CP2)	7	3	2
SAE (PO3)	6	4	2	SAE (P4)	7	4	2
SAE (O1)	7	5	2	SAE (P8)	6	4	3
SAE (Oz)	6	3	3	SAE (PO4)	8	4	2
SAE (Pz)	8	6	2	SAE (O2)	7	4	2

**Table 3:** Accuracy comparison for combination of classifiers and feature extraction methods.

*(a) Valence*				
*Feature extraction method*				

Classifier type	Accuracy (%)	PCA	NPCA	KLD
	SVM	75.45	78.04	77.51
	KNN	74.81	76.42	76.05
	BN	75.32	77.41	76.13

*(b) Arousal*				
*Feature extraction method*				

Classifier type	Accuracy (%)	PCA	NPCA	KLD
	SVM	76.26	77.25	78.23
	KNN	73.45	74.91	75.63
	BN	74.96	75.56	76.91

**Table 4:** Computational time(s) to train for combination of classifiers and feature extraction methods.

*(a) Valence*				
*Feature extraction method*				

Classifier type	Time (s)	PCA	NPCA	KLD
	SVM	558	634	881
	KNN	452	841	847
	BN	593	729	1143

*(b) Arousal*				
*Feature extraction method*				

Classifier type	Time (s)	PCA	NPCA	KLD
	SVM	571	595	914
	KNN	470	537	914
	BN	623	755	1076

**Table 5:** Accuracy of SVM, BN, KNN, CapsNet, and CNN networks in image classification by ten features, including subband power, mean, standard deviation, zero-crossing rate, fractal dimension, entropy, and correlation dimension.

Classifiers	*Features*										
	Power theta	Power alpha	Power beta	Power gamma	Mean	Standard deviation	Zero-crossingrate	Fractal dimension	Approximate entropy	Correlation dimension	SAETM
SVM	0.5132 ± 0.02	0.5818 ± 0.01	0.4363 ± 0.06	0.5527 ± 0.01	0.3280 ± 0.13	0.3620 ± 0.02	0.4750 ± 0.12	0.5145 ± 0.03	0.4239 ± 0.05	0.3840 ± 0.01	0.7536 ± 0.01
BN	0.4746 ± 0.13	0.5373 ± 0.02	0.5248 ± 0.05	0.4323 ± 0.01	0.4129 ± 0.01	0.3359 ± 0.01	0.3984 ± 0.03	0.4719 ± 0.11	0.3487 ± 0.15	0.4602 ± 0.04	0.6906 ± 0.12
KNN	0.5601 ± 0.02	0.4982 ± 0.12	0.4880 ± 0.05	0.3760 ± 0.05	0.3717 ± 0.01	0.3129 ± 0.04	0.4573 ± 0.04	0.3985 ± 0.03	0.4604 ± 0.04	0.4228 ± 0.02	0.7158 ± 0.04
CNN	0.6534 ± 0.03	0.6710 ± 0.04	0.5730 ± 0.07	0.5915 ± 0.04	0.4872 ± 0.06	0.3916 ± 0.01	0.4716 ± 0.02	0.5610 ± 0.04	0.5201 ± 0.07	0.5072 ± 0.12	0.8305 ± 0.02
CapsNet	0.6721 ± 0.06	0.6430 ± 0.11	0.5928 ± 0.02	0.6592 ± 0.07	0.5340 ± 0.16	0.4924 ± 0.12	0.5935 ± 0.04	0.6026 ± 0.15	0.5873 ± 0.02	0.6453 ± 0.13	0.8159 ± 0.01
Average (ACC)	0.5747 ± 0.052	0.5863 ± 0.06	0.5230 ± 0.05	0.5223 ± 0.036	0.4268 ± 0.074	0.3790 ± 0.04	0.4792 ± 0.05	0.5097 ± 0.072	0.4681 ± 0.066	0.4839 ± 0.064	0.7613 ± 0.04

The article "Extracting a Novel Emotional EEG Topographic Map Based on a Stacked Autoencoder Network" was published in 2023. Journal: J Healthc Eng.

**Table 6:** CNN network accuracy in image classification after 10 minutes for SAETM features and ten other features.

Time (m)	*Features*										
	Power theta	Power alpha	Power beta	Power gamma	Mean	Standard deviation	Zero-crossingrate	Fractal dimension	Approximate entropy	Correlation dimension	SAETM
1	0.4281	0.4323	0.4303	0.4183	0.4065	0.3619	0.4003	0.4549	0.4426	0.4273	0.4874
2	0.4170	0.4382	0.4580	0.4089	0.4103	0.3547	0.4097	0.4609	0.4432	0.4175	0.4787
3	0.4295	0.4693	0.4531	0.4198	0.4074	0.3683	0.4162	0.4656	0.4594	0.4145	0.5996
4	0.4536	0.4726	0.4854	0.4186	0.4238	0.3605	0.4229	0.4768	0.4529	0.4291	0.6491
5	0.4609	0.4812	0.4930	0.4347	0.4239	0.4038	0.4140	0.4611	0.4535	0.4043	0.7752
6	0.4729	0.4983	0.5034	0.4279	0.4158	0.3794	0.4371	0.4662	0.4485	0.4296	0.7923
7	0.4582	0.4978	0.5012	0.4376	0.4283	0.3775	0.4395	0.4693	0.4526	0.4352	0.8164
8	0.4901	0.5391	0.5078	0.4594	0.4192	0.3738	0.4588	0.4738	0.4594	0.4808	0.8283
9	0.5865	0.6449	0.5539	0.5523	0.4763	0.3875	0.4521	0.5532	0.4820	0.4986	0.8298
10	0.6534	0.6710	0.5730	0.5915	0.4872	0.3916	0.4716	0.5610	0.5201	0.5072	0.8305

## Data Availability

The DEAP Dataset (A Dataset for Emotion Analysis) used to support the findings of this study were supplied by Sander Koelstra et al. under license and so cannot be made freely available. Requests for access to these data should be made to (i.patras@eecs.qmul.ac.uk, https://www.eecs.qmul.ac.uk/mmv/datasets/deap/).
